# Evaluation of the Property of Axillary Lymph Nodes and Analysis of Lymph Node Metastasis Factors in Breast Cancer by Ultrasound Elastography

**DOI:** 10.1155/2022/8066289

**Published:** 2022-06-03

**Authors:** Jia Zhou, Qingyu Zhang, Qi Zhang, Lei Yan, Qing Gao

**Affiliations:** ^1^Department of Ultrasonic, The Second Affiliated Hospital of Mudanjiang Medical University, Mudanjiang 157009, China; ^2^Department of Anesthesiology, The Second Affiliated Hospital of Mudanjiang Medical University, Mudanjiang 157009, China; ^3^Department of Histology and Embryology, Mudanjiang Medical University, Mudanjiang 157011, China; ^4^Clinical Skills Center of The First Clinical College, Mudanjiang Medical University, Mudanjiang 157011, China

## Abstract

This research was aimed at investigating the role of ultrasound elastography (UE) in evaluating the properties of axillary lymph nodes in breast cancer and exploring the influencing factors of lymph node metastasis in breast cancer patients. Routine ultrasonography (US) and UE were performed for 160 breast cancer patients. 80 cases were in the group with lymph node metastasis, and the other 80 were in the nonlymph node metastasis group. The sensitivity, specificity, and accuracy of the two ultrasound examinations were compared, the receiver-operator characteristic (ROC) curves were drawn, and the influencing factors of lymph node metastasis were analyzed. The sensitivity, specificity, and accuracy of UE in diagnosing axillary lymph nodes of breast cancer were 97.22%, 95.45%, and 96.25%, respectively, which were markedly higher than those of routine US (*P* < 0.05). Cortical thickness, blood flow grade, blood flow type, and elasticity score had a greater impact on axillary lymph node metastasis of breast cancer. When cortical thickness ≥ 3 cm, blood flow was of 2-3 grades, blood flow was the peripheral/mixed type, and elasticity score was 3-4 points, these became risk factors for lymph node metastasis in breast cancer patients. UE was effective in diagnosing the property of lymph nodes and could evaluate lymph node metastasis in breast cancer patients. It had a good clinical value and was worthy of popularization and application.

## 1. Introduction

Breast cancer is one of the tumors that seriously affects women's health, with a high incidence and a younger population [1]. Compared with that in western developed countries, the incidence of breast cancer in China is relatively lower. However, the incidence of breast cancer still ranks first among those of female malignant tumors in China [2]. The etiology of breast cancer is complex and is affected by environmental and own factors, of which hereditary and hormone levels are important influencing factors [3]. The symptoms of early breast cancer are atypical and often overlooked. Breast cancer is mostly found during physical examination, and it is usually in the middle and late stages when it is discovered [4]. The metastasis of axillary lymph nodes is an important factor to evaluate the overall survival (OS) and disease-free survival (DFS) of breast cancer patients. It is positive to investigate the property of axillary lymph nodes in breast cancer and the influencing factors of lymph node metastasis, which can provide the clinical reference for the treatment of breast cancer [5]. In addition, knowing whether the patient has axillary lymph node metastasis before surgery has a guiding significance for the selection of surgical methods and formulation of treatment plans [6].

Ultrasonography (US) is a common method for determining the properties of axillary lymph nodes and lymph node metastases of breast cancer [7]. Doppler ultrasound has the advantages of convenient operation, noninvasive safety, and high acceptance of patients, having a good clinical application effect in the property determination and metastasis analysis of axillary lymph nodes [8–10]. Ultrasound elastography (UE) is a new ultrasound examination technology that has been gradually applied in clinical examinations. UE can image different deformation degrees of tissues with different hardness coefficients after being compressed by external forces. It is usually used for the detection of lesions that cannot be detected by routine US. The elastic images are shown in green for tissues with medium elastic coefficient, in red for tissues with large displacement after compression, and in blue for tissues with small displacement after compression. It can assess the deformability of tissues, show the tissue elasticity, and reflect the biological characteristics of lesions [11]. The elasticity of biological tissue depends on the molecular composition of the tissue. For malignant lesions, the internal structure of the tissue changes, and the elastic characteristics also change [12]. Ultrasound imaging combined with digital signal processing can get to know the internal displacement, strain, and other parameters of the tissue and reflect the difference of its elastic mechanical properties [13]. The strain of hard tissues is relatively smaller, and the strain of soft tissues is relatively greater [14]. At present, UE has been widely used in the diagnosis of breast, thyroid, liver, cervix, and lymph nodes, so it has become a practical auxiliary method for ultrasonic diagnosis [15].

The role of UE in the diagnosis of axillary lymph node properties and metastasis of breast cancer was explored in this work. The application value of two ultrasound methods in judging the lymph node properties in breast cancer patients was also investigated. The sensitivity, specificity, and accuracy of both routine US and UE were calculated in diagnosing the properties of axillary lymph nodes, and the risk factors for lymph node metastasis in breast cancer were analyzed. The objective and significance of this research was to provide the choice of examination methods for the judgment of lymph node properties and metastasis in breast cancer patients. Furthermore, a reference for the treatment and prevention of lymph node metastasis in breast cancer patients was also provided.

## 2. Materials and Methods

### 2.1. Research Objects

In this research, 160 patients with breast cancer admitted to hospital from January 2018 to December 2020 were selected as the research objects, all of whom were female. The included patients were divided into two groups, as 80 cases in metastatic lymph node group and 80 cases in nonmetastatic lymph node group. The general data of patients were shown in Table 1. All the patients included underwent routine US as well as UE to compare the diagnostic effects of different examination methods. The influencing factors of axillary lymph node metastasis of breast cancer were also researched. With no statistical difference in the general data of patients in the two groups, there was a comparability. All patients and their family members understood and signed informed consent. This study had been approved by the ethics committee of the hospital.

Inclusion criteria: the patients had complete medical records and imaging data; the patients had no other malignant tumors; those had not genetic diseases; those patients and their families signed informed consent.

Exclusion criteria: the patients got communication impairment; those were complicated with vital organ diseases; and those were unwilling to participate in.

### 2.2. Ultrasound Examinations

All patients in this research were examined by color ultrasonic instrument, and the probe frequency was set at 5.0-13.0 MHz. The patients were assisted in a supine position with the arms raised to expose the axilla. The patients should maintain steady breathing and first underwent a routine US examination. The axial ratio, cortical thickness, and blood flow of the patients' axillary lymph nodes were observed and recorded. Afterwards, the largest long-axis section was selected for the UE, and the elasticity scores of the axillary lymph nodes were recorded. The elastography mode was chosen for the ultrasonic instrument, and the probe was placed above the mass as well as perpendicular to the skin. The probe was slightly vibrated to obtain elastographic images of the region of interest. Elastography was assessed using ChoiJJ's 4-point method. If all the lymph nodes were green or a little blue, it was scored to be 1 point. 2 points meant there were scattered blue areas, with the proportion less than 45%. 3 points indicated that the blue areas were greater than 45%. If the blue area occupied the entire lymph nodes with or without green borders, it was scored as 4 points.

The pathological classification standards of breast tumors were in accordance with the histological classification and diagnostic criteria of breast tumors by World Health Organization.

### 2.3. Observation Indicators

The number of cases with benign and malignant axillary lymph nodes were counted through pathological examination, routine US, and UE.

The sensitivity, specificity, and accuracy of routine US and UE were calculated in diagnosing the property of axillary lymph nodes. The calculation method of the sensitivity of routine US was shown as Equation (1), that of specificity was shown as Equation (2), and that of accuracy was as Equation (3). For UE, the calculation method of the sensitivity, specificity, and accuracy was expressed as Equations (4), (5), and (6), respectively. In these equations, PB represented the number of patients with benign pathology, and PM was the number of patients with malignant pathology. USB referred to the number of benign patients diagnosed with routine US, while USM was the number of malignant patients under routine US. UEB was the number of pathologically benign patients under UE, and UEM was the number of pathologically malignant patients under UE.

(1) $$\begin{array}{c} {\text{Sensitivity}}_{\text{US}}=\frac{\text{USM}}{\text{PM}}, \end{array}$$

(2) $$\begin{array}{c} {\text{Specificity}}_{\text{US}}=\frac{\text{USB}}{\text{PB}}, \end{array}$$

(3) $$\begin{array}{c} {\text{Accuracy}}_{\text{US}}=\frac{\text{USM}+\text{USB}}{\text{PB}+\text{PM}}, \end{array}$$

(4) $$\begin{array}{c} {\text{Sensitivity}}_{\text{UE}}=\frac{\text{UEM}}{\text{PM}}, \end{array}$$

(5) $$\begin{array}{c} {\text{Specificity}}_{\text{UE}}=\frac{\text{UEB}}{\text{PB}}, \end{array}$$

(6) $$\begin{array}{c} {\text{Accuracy}}_{\text{UE}}=\frac{\text{UEM}+\text{UEB}}{\text{PB}+\text{PM}}. \end{array}$$

The receiver-operator characteristic (ROC) curves of the two ultrasound methods were drawn for diagnosing the property of axillary lymph nodes.

The influencing factors of axillary lymph node metastasis of breast cancer were analyzed. The main influencing factors included the axial ratio, cortical thickness, blood flow grades, blood flow types, blood flow resistance, and elasticity score. In the two groups, the numbers of patients with long-short axial ratio < 2 and that ≥2 were counted. The number of patients with cortical thickness ≥ 3 cm and that <3 cm, the number of patients with blood flow in grade 0-1 and that with grade 2-3, as well as the number of patients with no-flow/portal type and that with peripheral/mixed type were also counted. Besides, the number of people with blood flow resistance ≥ 0.6 and that <0.6, and the number of patients whose elasticity score was in 1-2 points and that in 3-4 points were counted, respectively.

### 2.4. Statistical Methods

SPSS 20.0 was used for statistical analysis of data, the ROC curves were drawn, and *t*-test was adopted. The enumeration data were expressed by rate (%), and it was considered that *P* < 0.05 indicated a difference was of statistically significance.

## 3. Results

### 3.1. Comparison of Images of Lymph Node Metastasis of Breast Cancer in Different Ultrasound Types

Figure 1 displayed images comparing lymph node metastases in breast cancer under different ultrasonic types. Image A was under the routine US, while Image B was an image of UE. In the elastic image, green represented tissues with medium elastic coefficient, red was the tissues with large displacement after compression, and blue stood for tissues with small displacement after compression. It could be observed that UE was more intuitive and clearer, having better evaluation and diagnosis effects.

### 3.2. Comparison of Two Ultrasound Methods in Diagnosing the Property of Axillary Lymph Nodes

Table 2 displayed the comparison results of the two ultrasound methods in the diagnosis of the property of axillary lymph nodes. The results of pathological examination showed that there were 88 patients with benign axillary lymph nodes and 72 patients with malignant ones in total. Examined by routine US, 88 patients had benign axillary lymph nodes, of which 81 cases were diagnosed correctly. 72 malignant patients were detected out, of which 65 cases were examined with the correct results. By UE, there were a total of 86 benign patients, and 84 of them went with correct property; among 74 malignant patients, the results of 70 cases were correct.

### 3.3. Comparison of Two Ultrasound Methods in the Diagnosis Efficacy of Axillary Lymph Nodes

Figures 2–4 represented the comparison of the sensitivity, specificity, and accuracy of diagnosing the property of axillary lymph nodes. It was shown that the sensitivity of the diagnosis by UE was 97.22%, the specificity was 95.45%, and the accuracy was 96.25%. By routine US, the sensitivity, specificity, and accuracy were 90.28%, 92.05%, and 91.25%, respectively, in diagnosing the property of axillary lymph nodes. All the sensitivity, specificity, and accuracy of UE were higher than those of routine US, and the differences were statistically significant (*P* < 0.05).

### 3.4. ROC Curves of Two Ultrasound Methods in Diagnosing the Property of Axillary Lymph Nodes

The ROC curves of the two ultrasound methods were shown in Figure 5. It could be found that UE had a better diagnostic effect in diagnosing the property of axillary lymph nodes and also the better application effect.

### 3.5. Analysis of Influencing Factors of Axillary Lymph Node Metastasis in Breast Cancer

As shown in Figure 6, the influencing factors of axillary lymph node metastasis of breast cancer were analyzed. Figures 6(a)–6(f) showed the axial ratio of long and short axes, cortical thickness, blood flow grades, blood flow types, blood flow resistance, and elasticity score, respectively. The axial ratio, cortical thickness, blood flow grade, blood flow type, blood flow resistance index, and elasticity score were all influencing factors of axillary lymph node metastasis in breast cancer. Among these influencing factors, cortical thickness had the greatest impact on axillary lymph node metastasis in breast cancer. It could be known from the figures that, among breast cancer patients without axillary lymph node metastasis, the cortical thickness of 50 cases was <3 cm, and that ≥3 cm in 30 cases. Among the patients with lymph node metastasis, 4 cases had the cortical thickness < 3 cm, while 76 cases had that ≥3 cm. Thus, the cortical thickness in breast cancer patients with axillary lymph node metastasis was thicker, and most of the patients got a cortical thickness ≥ 3 cm.

## 4. Discussion

The earliest metastasis route of breast cancer is the axillary lymph node metastasis. Whether a patient has axillary lymph node metastasis is an important basis for judging the clinical stage and formulating a treatment plan for the patient [16]. The metastasis of axillary lymph nodes is also an important indicator to evaluate the recovery and development trend of breast cancer patients [17]. The breasts are in front of the chest and bulge forward, with very rich lymphatic drainage. There are abundant lymphatic vessels under the breast skin and under the nipples [18]. Most of the lymph flow from the outside of the breasts to the anterior thoracic lymph nodes and then to the axillary lymph nodes [19]. Breast cancer patients with axillary lymph node metastasis are very likely to relapse, and the risk of distant metastasis is also greatly increased, which is not conducive to the prognosis and disease recovery [20]. Lymph node metastasis usually occurs when the tumor's diameter increases, the number of lymph node metastases would increase, and the disease continues to deteriorate [21]. With the development of modern medical equipment technology, preliminary diagnosis and classification of disease has become a common method. Ultrasound diagnosis is a widely used method, which is highly accepted by patients, easy to apply, and with significant effects, having been unanimously recognized by patients and doctors [22]. The diagnostic value of two ultrasound methods was explored for the property and metastasis of axillary lymph nodes in breast cancer, the effect of UE in diagnosing the property of axillary lymph nodes was investigated, and the risk factors affecting lymph node metastasis in breast cancer were analyzed.

Axillary lymph node metastasis is a common marker of deterioration in breast cancer patients; therefore, the diagnosis and evaluation of axillary lymph nodes is an important examination for breast cancer patients. Among the 160 patients included, 88 cases had benign axillary lymph nodes and 72 cases got malignant axillary lymph nodes. There is a high probability of false negatives in routine US, and the accuracy of the examination needs to be improved [23]. UE is a newly developed ultrasound examination method, which is efficient, accurate, and less invasive with a high application value [24]. UE is helpful for doctors to grasp the property and metastasis of axillary lymph nodes in patients, judge the disease stage of patients, and give patients appropriate treatment plans [25]. Some studies have found that compared with routine US, the new method of UE has the better sensitivity, specificity, and accuracy in the diagnosis of breast tumors [26]. Han et al. (2018) [27] found that in the qualitative diagnosis of breast cancer, UE could diagnose the disease more accurately and could be used in clinical practice successfully. Wang et al. (2020) [28] found that UE had a high value in predicting the treatment effect of breast cancer. This research also found that 81 benign patients detected by routine US had correct results, and 65 malignant patients detected went with the correct results. 84 benign patients detected by UE had correct results, while 70 malignant patients detected got the correct results. The accuracy of UE in diagnosing the property of axillary lymph nodes was higher than that of routine US. The sensitivity, specificity, and accuracy of UE in diagnosing the property of axillary lymph nodes were 97.22%, 95.45%, and 96.25%, respectively, while that of routine US were 90.28%, 92.05%, and 91.25%, respectively. The sensitivity, specificity, and accuracy of UE in diagnosing the property of axillary lymph nodes were all higher than those of routine US.

It was suggested that compared with routine US, UE had a better effect in diagnosing the property of axillary lymph nodes. Ultrasonographic axial ratio, cortical thickness, blood flow grades, blood flow types, blood flow resistance index, and elasticity score were all influencing factors of axillary lymph node metastasis in breast cancer. Cortical thickness, blood flow grades, blood flow types, and elasticity score had the greater impact on axillary lymph node metastasis of breast cancer. Breast cancer patients with cortical thickness ≥ 3 cm, blood flow grade 2-3, peripheral/mixed blood flow type, and elasticity score of 3-4 points were more likely to suffer from lymph node metastasis. UE could improve clinical guidance for the diagnosis of breast cancer patients, the judgment of lymph node properties, and the evaluation of metastasis.

## 5. Conclusion

It was found that UE had a higher value in evaluating the properties and metastasis of axillary lymph nodes in breast cancer. UE had the higher sensitivity, specificity, and accuracy than routine US. For UE was simple to operate and had a great evaluation effect, it could be applied to the clinical judgment of lymph node properties in breast cancer patients, showing a positive significance. The main risk factors for lymph node metastasis in breast cancer included axial ratio, cortical thickness, blood flow grade, blood flow type, blood flow resistance index, and elasticity score. The disadvantage of this research was that the sample size was small, so further proofs of the results were required.

## Figures and Tables

**Figure 1:** Comparison of lymph node metastases of breast cancer in different ultrasound methods. (a) Routine US; (b) UE.

**Figure 2:** Comparison of the sensitivity of two ultrasonic methods in diagnosing the properties of axillary lymph nodes. ^∗^Compared with the nonlymph node metastasis group, *P* < 0.05.

**Figure 3:** Comparison of the specificity in the diagnosis of axillary lymph node properties between two ultrasonic methods. ^∗^Comparison with the nonmetastatic lymph node group, *P* < 0.05.

**Figure 4:** Comparison of the accuracy in determining the properties of axillary lymph nodes between two types of ultrasounds. ^∗^Compared with the group of nonmetastatic lymph node, *P* < 0.05.

**Figure 5:** ROC curves of two ultrasound methods in diagnosing the property of axillary lymph nodes.

**Figure 6:** Analysis of influencing factors of axillary lymph node metastasis in breast cancer. (a) represented the axial ratio of long and short axes, (b) was cortical thickness, (c) was blood flow grades, (d) was blood flow type, (e) was blood flow resistance index, and (f) was elasticity score. ^∗^Compared with the group of nonmetastatic lymph node, *P* < 0.05.

**Table 1:** Comparison of general data between the two groups of patients.

	Age	Medical history
Metastatic lymph node	38.67 ± 5.53	5.78 ± 1.98
Nonmetastatic lymph node	37.92 ± 5.78	5.96 ± 1.86

**Table 2:** Comparison of the property of axillary lymph nodes by two ultrasound methods.

Ultrasound examinations		Pathological examination	
		Malignant	Benign
Routine US	Malignant	65	7
	Benign	7	81
UE	Malignant	70	4
	Benign	2	84

## Data Availability

The data used to support the findings of this study are available from the corresponding author upon request.
